The article "Metabolism of 2-Chloro-4-Nitroaniline via Novel Aerobic Degradation Pathway by Rhodococcus sp. Strain MB-P1" was retracted in 2014. Reasons: fabricated or falsified data; fabricated or falsified results.

# Metabolism of 2-Chloro-4-Nitroaniline via Novel Aerobic Degradation Pathway by *Rhodococcus* sp. Strain MB-P1

**DOI:** 10.1371/journal.pone.0062178

**Published:** 2013-04-17

**Authors:** Fazlurrahman Khan, Deepika Pal, Surendra Vikram, Swaranjit Singh Cameotra

**Affiliations:** Institute of Microbial Technology, Council of Scientific and Industrial Research (CSIR), Chandigarh, India; University of Kansas, United States of America

## Abstract

2-chloro-4-nitroaniline (2-C-4-NA) is used as an intermediate in the manufacture of dyes, pharmaceuticals, corrosion inhibitor and also used in the synthesis of niclosamide, a molluscicide. It is marked as a black-listed substance due to its poor biodegradability. We report biodegradation of 2-C-4-NA and its pathway characterization by *Rhodococcus* sp. strain MB-P1 under aerobic conditions. The strain MB-P1 utilizes 2-C-4-NA as the sole carbon, nitrogen, and energy source. In the growth medium, the degradation of 2-C-4-NA occurs with the release of nitrite ions, chloride ions, and ammonia. During the resting cell studies, the 2-C-4-NA-induced cells of strain MB-P1 transformed 2-C-4-NA stoichiometrically to 4-amino-3-chlorophenol (4-A-3-CP), which subsequently gets transformed to 6-chlorohydroxyquinol (6-CHQ) metabolite. Enzyme assays by cell-free lysates prepared from 2-C-4-NA-induced MB-P1 cells, demonstrated that the first enzyme in the 2-C-4-NA degradation pathway is a flavin-dependent monooxygenase that catalyzes the stoichiometric removal of nitro group and production of 4-A-3-CP. Oxygen uptake studies on 4-A-3-CP and related anilines by 2-C-4-NA-induced MB-P1 cells demonstrated the involvement of aniline dioxygenase in the second step of 2-C-4-NA degradation. This is the first report showing 2-C-4-NA degradation and elucidation of corresponding metabolic pathway by an aerobic bacterium.

## Introduction

2-Chloro-4-nitroaniline (C_6_H_5_ClN_2_O_2_, 2-C-4-NA) is a nitroaromatic compound, used as an intermediate in the synthesis of dyes, pharmaceuticals, corrosion inhibitors and in the manufacture of niclosamide, a molluscicide [1]–[3]. 2-C-4-NA is also reported as a photolysis product of niclosamide [4]. Espinosa-Aquirre et al. [5] reported the metabolism of niclosamide, which is used as an anti-helminthic drug, results in the formation of 2-C-4-NA and 5-chlorosalicylic acid metabolites by hydrolytic cleavage of amide bond. As a result of its extensive production and application it may get released into the environments through various waste streams and is considered to be an increasing threat into the environments and various life forms [6]. Hence the fate of 2-C-4-NA in the environments is of great concern. 2-C-4-NA causes severe cellular damage as studied in rat [7]. It is identified as a bacterial mutagenic compound as tested in *Salmonella typhimurium*, however, the potency is low compared to niclosamide [5]. The environmental fate of 2-C-4-NA can be determined either by non-biological (volatization, hydrolysis, photolysis, thermal decomposition) or by biological means. Volatization of 2-C-4-NA from the soil surface and water surface are not considered to be an important fate process owing to its Henry's Law constant of 9.5×10^−9^ atm-cu m mole^−1^ [8]. Similarly, 2-C-4-NA does not contain any functional group by which it would hydrolyze in the environment [9]. However, 2-C-4-NA contain chromophores that can absorb light at wavelength of >290 nm and may be susceptible to photolysis [9]. Thus, for the remediation of the heavy contamination in the environment, the microbial transformation and degradation could be used as the most effective, eco-friendly and technically challenging approach for the decontamination of soil, sediment and water bodies etc. 2-C-4-NA is considered to be non-biodegradable in the aquatic environment as well as in the industrial sewage treatment plants [10]. Similarly, Canton et al. [11] also classified 2-C-4-NA as a blacklist substance due to its poor biodegradability. However, based on the previous reports on the biodegradation of structural analogues of 2-C-4-NA such as 4-nitroaniline, 2-, 3-, 4-chloroaniline and 3, 4-dichloroaniline, possibilities for the biodegradation of 2-C-4-NA by microorganisms could also be presumed [12]–[18]. In this communication, we report metabolic characterization of 2-C-4-NA by *Rhodococcus* sp. strain MB-P1 which was previously characterized for the degradation of atrazine. The strain MB-P1 was capable of metabolizing 2-C-4-NA as the sole carbon, nitrogen, and energy source. The catabolic pathway for degradation of 2-C-4-NA by strain MB-P1 is initiated via oxidative hydroxylation resulting in the formation of 4-A-3-CP. Subsequent degradation occurs by dioxygenase mediated transformations as indicated by detection of ‘6-chlorohydroxyquinol’ (6-CHQ) as the terminal aromatic intermediate. This study has significant implications in terms of understanding the mechanism of aerobic degradation of 2-C-4-NA, related aromatic amines as well as determining their environmental fate.

## Materials and Methods

### Chemicals, strain, and growth medium

Analytical grade of 2-chloro-4-nitroaniline (2-C-4-NA) and standard 4-amino-3-chlorophenol (4-A-3-CP) were purchased from Sigma-Aldrich (St, Louis, MO, USA). *Rhodococcus* sp. strain MB-P1 was isolated from the contaminated soil sample and characterized for atrazine degradation [19]. Minimal salt medium (MSM) used in the present study was prepared as described earlier [19] with slight modification i. e. absence of nitrogen source [(NH_4_)_2_SO_4_]. Stock solution (10 mM) of 2-C-4-NA prepared in HPLC grade methanol was added to an empty Erlenmeyer flask to obtain the working concentrations. Further, the residual methanol in the flask was evaporated under a stream of air to leave the dry crystal of 2-C-4-NA in the bottom of the flask. Appropriate volume of MSM was added to the flask to attain desired working culture. Nutrient agar at one-quarter strength (1/4-NA) and nutrient broth (1/4-NB) were used as a rich media for bacterial growth and culture maintenance.

### Metabolic activity of strain MB-P1 on 2-C-4-NA

Metabolic activity of strain MB-P1 on 2-C-4-NA was determined by growth studies carried out in carbon-free MSM supplemented with varying concentrations of 2-C-4-NA ranging from 50 to 500 µM. The positive metabolic activity was determined by time dependent bacterial growth measure in terms of increase in optical density of the culture medium monitored at 600 nm using Lambda EZ 201 UV-visible spectrophotometer (Perkin-Elmer Inc, USA). Bacterial growth was also monitored by measuring the total protein of the cultures grown on 2-C-4-NA with Pierce BCA protein assay kit (Thermo Scientific, USA). Release of nitrite ions (NO_2_^−^), chloride ions (Cl^−^), and ammonia (NH_3_) in the growth medium and gradual decrease in concentration of 2-C-4-NA were monitored as the alternative methods for determination of metabolic activity of strain MB-P1 on 2-C-4-NA. Subsequent characterization was carried out to determine the kinetics of 2-C-4-NA degradation by strain MB-P1. Appropriate biotic and abiotic controls were included wherever necessary. Procedures used for growth studies and resting cell studies are as follows:

### Growth studies

Growth studies were performed in 50 ml of carbon-free MSM supplemented with 2-C-4-NA (200 µM) by inoculating 1% (v/v) of overnight culture of MB-P1 cells grown in 1/4-NB. Cultures were incubated on a rotary shaker at 200 rpm at 30°C. Samples were withdrawn at every 8 h to monitor bacterial cell growth, release of NO_2_^−^, Cl^−^, NH_3,_ and degradation of the growth substrate. Cell growth was monitored spectrophotometrically as described above. Bacterial growth was also monitored by the indirect approach of measuring total protein concentration in the culture. Culture fluid samples (2.0 ml) were centrifuged at 8,000×g for 10 min to obtain cell-free culture supernatants that were subsequently analyzed for NO_2_^−^, Cl^−^, and NH_3_ release, depletion of growth substrate and identification of degradation intermediates using methods described later. Non-inoculated flask and flask inoculated with heat killed cells of strain MB-P1 were used as abiotic control and negative control respectively.

### Resting cell studies

Resting cell studies were performed with minor modification of the method described earlier [20]. Briefly, a seed culture (6%, v/v) of strain MB-P1 grown in 1/4-NB inoculated into 1.6 L of 1/4-NB supplemented with 200 µM of 2-C-4-NA and incubated at 30°C with aeration for 24 h (OD_600_, 1.3–1.4). The induced cells were harvested by centrifugation at 8,000×g at room temperature for 10 minutes, washed twice with phosphate buffer (20 mM, pH 7.2) and suspended in 100 ml of carbon-free MSM. This suspension was divided into four aliquots of 25 ml each; one aliquot was heat killed by incubating on boiling water for 30 minutes which was later used as negative control. The other two aliquots were supplemented with 200 µM of 2-C-4-NA and 4-A-3-CP separately. Each flask was then incubated at 30°C with shaking at 200 rpm. Similarly, another control for the above experiment was also made by suspending un-induced cells of strain MB-P1 in MSM supplemented with 200 µM of 2-C-4-NA and 4-A-3-CP separately. Samples (2.0 ml) were withdrawn from both control and experimental flasks at regular intervals of 2 h and subjected to NO_2_^−^, Cl^−^, and NH_3_ release analysis, followed by high-performance liquid chromatography (HPLC) analysis and also gas chromatography-mass spectroscopy (GC-MS) analyses (methods described later).

### Ring cleavage inhibition studies

There is a well known study to check the inhibition of ring cleavage catalyzed by ferrous ions dependent ring cleavage dioxygenase by using an iron chelator i. e. 2, 2-dipyridyl [21]. The ring cleavage experiment was performed in the same way as the resting cell study. The harvested 2-C-4-NA-induced resting cells were suspended in 25 ml carbon-free MSM supplemented with 200 µM of 2-C-4-NA and 1.0 mM 2, 2-dipyridyl. Similarly, another flask was also taken as a control containing 25 ml cell suspensions of 2-C-4-NA-induced resting cells in MSM supplemented with 200 µM of 2-C-4-NA only. Each flask was then incubated at 30°C with shaking at 200 rpm. Culture supernatant (2.0 ml) was collected at different time intervals and analyzed by HPLC.

### Enzyme assays with cell-free lysates

2-C-4-NA-induced cells of strain MB-P1 were harvested by centrifugation and were washed twice with phosphate buffer (20 mM, pH 7.2) and finally re-suspended in lysis buffer (50 mM phosphate buffer, pH 7.2). Cell lysis was carried out by two passages through a French pressure cell (20,000 lb/in^2^). The lysed cell suspensions were centrifuged at 12,000 rpm for 30 min at 4°C and supernatant was carefully separated to obtain cell-free enzyme extract, which was subsequently used for the enzyme assays. Quantitation of protein content within cell-free extracts were performed routinely with Pierce BCA protein assay kit (Thermo Scientific, USA). The cell-free extract was tested for activity of monooxygenase since this enzyme is known to be involved in the first step of 2-C-4-NA degradation as indicated by the identification of the pathway metabolites. The monooxygenase enzyme assay was carried out as described below:

### Enzyme assays for monooxygenase

Flavin-dependent monooxygenase enzyme activity was assayed to characterize the putative first step of 2-C-4-NA degradation by strain MB-P1. Cell-free protein extracts (5 mg ml^−1^ of protein) prepared from 2-C-4-NA-induced cells were added to phosphate buffer (20 mM, pH 7.0), 100 µM NADPH, 200 µM FMN in a total reaction volume of 10 ml. Reactions were initiated by the addition of 70 µM 2-C-4-NA and incubated at 28°C. Samples were withdrawn at regular time intervals and monooxygenase enzyme activity was determined by measuring the time dependent disappearance of 2-C-4-NA and NO_2_^−^ release. The 2-C-4-NA depletion was measured by HPLC analysis. Release of NO_2_^−^ ions were estimated with the colorimetric method described later.

### Enzyme assay for aniline dioxygenase

The aniline dioxygenase enzyme activity by strain MB-P1 was measured with an oxygen electrode (YSI, Ohio, USA), according to the method described by Liu et al. [22]. MB-P1 cells grown in 500 ml 1/4-NB were harvested by centrifugation at 8,000×g at 4°C for 10 minutes. Pellets were washed twice with phosphate buffer (20 mM, pH 7.2) and suspended in 100 ml of MSM containing 2-C-4-NA (100 µM). In order to obtain the un-induced cells, the similar cell pellets were suspended in 100 ml of 1/4-NB. Further, these cells were incubated at 30°C under shaking at 200 rpm to obtain 2-C-4-NA-induced or non-induced cells respectively. After 24 h of incubation, cells were harvested, cell pellets were washed twice with phosphate buffer (20 mM, pH 7.2) and re-suspended in the same buffer. This suspension was used for the assay of aniline dioxygenase by measuring oxygen uptake at 30°C.

### Analytical methods

The release of nitrite ions (NO_2_^−^) was monitored with a colorimetric method using N-(1-naphthyl) ethylene-diamine-dihydrochloride and sulfanilic acid reagent as described earlier [23]. Ammonia (NH_3_) concentrations were also monitored with a colorimetric method using ‘Ammonia Estimation Kit’ (Sigma Aldrich, USA) according to the manufacturers' recommendation. Similarly, the release of chloride ions (Cl^−^) was also monitored colorimetrically with colorimetric method that uses mercuric thiocyanate [24]. Standard plots generated with known concentrations of NaCl, (NH_4_)_2_SO_4_ and NaNO_2_ were used to determine the concentrations of Cl^−^, NH_4_^+^, and NO_2_^−^ ions released into the culture medium.

For the quantitative measurement of 2-C-4-NA degradation by strain MB-P1 and identification of metabolic products, 500 µl of cell-free aqueous culture supernatants from growth and resting cell studies were filtered with 0.2 µm filters (Millipore Inc. USA). The filtered culture supernatants were analyzed with minor modification of the quantitative HPLC method described earlier [25]. Briefly, the separation of 2-C-4-NA and their metabolic products was carried out on a C-18 reverse phase column at 30°C on UV-detector equipped Waters HPLC system (Waters, USA). The mobile phase used was a mixture of acetonitrile:water (30∶70, v/v) under an isocratic condition with the flow rate of 1.0 ml min^−1^. The peaks of analytes were detected with UV detector over a wavelength scan of 220–290 nm. Alternatively for the analysis of metabolites by GC-MS, cell-free aqueous culture supernatant samples were mixed with equal volume of ethyl acetate and performed liquid-liquid extraction by layer separation sequentially at neutral and acidic pH. Extracted organic phase was pooled, dried under nitrogen flow using RotaVapor II (BUCHI, Switzerland) and re-suspended in the appropriate volumes of ethyl acetate. The derivatization of metabolic products in the sample was performed by silylation as previously described [26]. The derivatized samples were analyzed by GC-MS using QP2010S (Shimadzu Scientific Instruments, USA) with temperature program and run parameter used for GC analyses as reported earlier [27]. Briefly, temperature program was: 1 min at 50°C, followed by ramping up to 150°C at a constant temperature increment rate of 20°C min^−1^, a slower ramping to 200°C at a rate of 5°C min^−1^, and then further ramped to 320°C at a rate of 20°C min^−1^, which was held for 5 min. Positive molecular ion mass spectra were scanned in mass/charge (m/z) range of 50–500.

## Results

### Growth study and degradation of 2-C-4-NA by strain MB-P1

Initial screening for the metabolic activity on 2-C-4-NA was carried out by using lab isolates (previously isolated from contaminated soil). A total 79 bacterial isolates were selected and screened for 2-C-4-NA degradation by inoculating in carbon-free MSM supplemented with 2-C-4-NA (100 µM). Thereafter 2-C-4-NA degrading abilities were examined by analyzing the growth of culture and release of NO_2_^−^, Cl^−^ ions, and NH_3_ in the medium. Five isolates showed apparent increase in bacterial cell mass and also the release of NO_2_^−^, Cl^−^ ions, and NH_3_. Among these isolates, strain MB-P1 was found to be an efficient degrader of 2-C-4-NA. The strain MB-P1 was incubated in carbon-free MSM supplemented with the different concentrations of 2-C-4-NA ranging from 50 to 500 µM. Noticeably complete inhibition of growth was observed when 2-C-4-NA was used at concentrations higher than 300 µM. However, 200 µM served as optimal concentration for growth of strain MB-P1 (data not shown). The growth study of strain MB-P1 carried out in carbon-free MSM supplemented with 2-C-4-NA (200 µM) showed an evident lag phase of 16 h (Figure 1). However, over time of subsequent log phase, the bacterial culture grew exponentially as observed with the increase of total protein concentration up to the value of 9.1 µg ml^−1^ (Figure 1). During the growth study, no metabolic products were detected from the sample analyzed by HPLC. However, NH_3_, Cl^−^ ions, and NO_2_^−^ ions released in the culture media were quantified colorimetrically. The released NH_3_ and NO_2_^−^ ions were quantified colorimetrically to be 30 µM and 198.5 µM respectively at the end of the log phase of the growth (Figure 1). The accumulation of lesser amount of NH_3_ in the media clearly suggested that NH_3_ was used as a preferred nitrogen source for its growth. On the other hand, Cl^−^ ions continued to accumulate in culture medium and reached a maximum concentration of 198.8 µM. The quantitative measurement of 2-C-4-NA by HPLC from growth medium showed its decrease from initial concentration of 200 µM to non-detectable amounts after∼90 h of incubation (Figure 1). The growth yield of strain MB-P1 on 2-C-4-NA was found to be 0.50 g of cells/g of 2-C-4-NA. Similarly, the rate of 2-C-4-NA degradation by strain MB-P1 during the growth studies was calculated to be 3.2 µmol mg protein^−1^ minute^−1^. The strain MB-P1 also utilized 4-A-3-CP as the sole carbon, nitrogen, and energy source with slight accumulation of NH_3_ (28 µM) in the culture media (Data not shown). The growth yield of strain MB-P1 on 4-A-3-CP was 0.62 g of cells/g of 4-A-3-CP and the rate of 4-A-3-CP degradation by strain MB-P1 was 3.0 µmol mg protein^−1^ minute^−1^. The growth yield of strain MB-P1 on 4-A-3-CP as well as the rate of 4-A-3-CP degradation was found almost similar as determined for 2-C-4-NA.

**Figure 1:** Growth characterization of *Rhodococcus* sp. strain MB-P1 on 2-C-4-NA as the sole carbon, nitrogen, and energy source. (•), 2-C-4-NA; (▴), NO_2_^−^; (Δ), NH_4_^−^; (○), Cl^−^; (▪), total protein. Values are presented as arithmetic means of data obtained from experiments carried out in triplicates; error bars represent standard deviation.

### Elucidation of catabolic pathway for 2-C-4-NA degradation by strain MB-P1

#### Resting cell studies

During the growth study we could not identify any putative metabolites of 2-C-4-NA metabolism. Therefore, samples from resting cell studies and enzyme assays were used for the identification of intermediates. The aqueous sample collected at different time intervals from the resting cell studies was analyzed by HPLC. The resting cell study showed that the induced cells eliminate the lag phase for the depletion of 2-C-4-NA with transient accumulation of 4-A-3-CP metabolite, which subsequently depleted over the time of incubation (Figure 2A). However, when the same 2-C-4-NA-induced cells were also incubated with 4-A-3-CP, there was a shorter induction period for the disappearance of 4-A-3-CP in the first phase which underwent faster depletion over the time of incubation, suggesting that the enzyme responsible for the degradation of 4-A-3-CP is inducible in nature (Figure 2B). Noticeably, lesser amount of 6-CHQ metabolite was also identified, which disappeared over time of incubation (Figure 2). The above two metabolites identified in HPLC showed retention time (R*t*) at 4.86 and 3.28 min respectively (Figure 3A). The R*t* value corresponding to the 4.86 min matched with the authentic standard of 4-A-3-CP. However, the R*t* value corresponding to the 3.28 min could not be characterized due to the non-availability of standard. Further, the confirmation and identification of unknown metabolites from the samples obtained from the resting cell study were subjected to mass fragmentation analysis by GC-MS. In GC-MS analysis two metabolic peaks appeared at R*t* values of 7.62 and 9.52 min respectively (Figure 3B). The mass fragmentation pattern for metabolite with a R*t* value of 7.62 min showed a conjugate ion at m/z value of 215 (representing silylated species: M^+^), 200 (M-CH_3_), 143, 73 [Si (CH_3_)_3_] (Figure 3C). The mass spectrum of this metabolite matched the known standard of 4-amino-3-chlorophenol. This metabolite would have probably resulted from direct denitrification of the aromatic nucleus without deamination. The second metabolite with a R*t* value of 9.52 min showed a conjugate ion at m/z value of 378, 376 (M^+^), 366, 361 (M-CH_3_), 288, 275, 273, 179, 73 [Si (CH_3_)_3_] (Figure 3C). The fragmentation pattern and mass spectra of this metabolite were consistent and similar to that of 6-chlorohydroxyquinol as described earlier [27]. 6-chlorohydroxyquinol is reported as the terminal intermediate in the degradation of 2, 4, 6-trichlorophenol and 2, 6-dichlorophenol degradation by *Azotobacter* sp. strain GP1, *Streptomyces rochei* 303, *Ralstonia eutropha* JMP 134 and *Cupriavidus necator* JMP134 [28]–[32]. The formation of 6-chlorohydroxyquinol metabolite would be as a result of dioxygenation with the deamination of amino group from the benzene ring. Based on the above, HPLC and GC-MS analysis, we conclude that 4-A-3-CP and 6-CHQ are the major identified metabolites during aerobic degradation of 2-C-4-NA by strain MB-P1.

**Figure 2:** Degradation kinetics of 2-C-4-NA and 4-A-3-CP during resting cell studies performed by 2-C-4-NA-induced cells of strain MB-P1. (A) 2-C-4-NA degradation kinetics. (•), 2-C-4-NA; (▪), 4-A-3-CP; (Δ), 6-CHQ; (○), 2-C-4-NA in abiotic control. (B) 4-A-3-CP degradation kinetics. (•), 4-A-3-CP; (Δ), 6-CHQ. Values are presented as arithmetic means of data obtained from experiments carried out in triplicates; error bars represent standard deviation.

**Figure 3:** Representative HPLC and GC-MS chromtograms along with mass spectra of metabolites identified during the degradation of 2-C-4-NA by resting cells of *Rhodococcus* sp. strain MB-P1. (A) HPLC chromatograms of metabolites identified at different time intervals. Peak at R*t* value of 8.5 min corresponds to 2-C-4-NA; Peak at R*t* value of 4.86 min corresponds to 4-A-3-CP; Peak at R*t* value of 3.28 min corresponds to 6-CHQ. (B) GC-MS chromatogram of the authentic standards and the identified metabolites. Peak at R*t* value of 6.41 min corresponds to 2-C-4-NA; Peak at R*t* value of 7.62 min corresponds to 4-A-3-CP; Peak at R*t* value of 9.52 min corresponds to 6-CHQ. (C) Mass spectra of metabolites (Left side; 4-A-3-CP and right side; 6-CHQ) of 2-C-4-NA as analyzed by GC-MS.

#### Enzyme assays

To validate the formation of metabolites and illustrate the degradation pathway of 2-C-4-NA in strain MB-P1, the enzyme assays were carried out. The formation of 4-A-3-CP as the first degradation metabolite and the release of NO_2_^−^ ions from 2-C-4-NA suggested oxygenase mediated enzymatic reaction in the degradation pathway. Cell lysates prepared from 2-C-4-NA grown cells of strain MB-P1 showed positive activity for flavin-dependent monooxygenase enzyme and catalyzed the elimination of NO_2_^−^ ions and formation of 4-A-3-CP. The specific activity for this enzymatic reaction was 1.3±0.25 nmol min^−1^ mg of protein^−1^.

#### Oxygen uptake

There was rapid oxygen consumption by 2-C-4-NA, 4-nitroaniline and 4-chloroaniline by 2-C-4-NA-grown cells (Table 1). The oxygen uptake of the above results showed that the pathway enzymes involved in the degradation of 2-C-4-NA are induced. However, the lesser amount of oxygen consumption by 2-C-4-NA by 1/4-NB grown cells revealed the first enzyme is constitutive in nature. Whereas, there was a negligible amount of oxygen uptake by aniline and 4-A-3-CP in 1/4-NB grown cells indicating inducible nature of the aniline dioxygenase. The above results are in close agreement with the results as reported earlier [22], [33], [34]. The NH_3_ released were also quantitatively measured and showed stoichiometry to the amount of substrates added (data not shown). Liu et al. [22] reported the formation of catechol product from aniline occurs via the action of aniline dioxygenase. Thus, based on the above results it is concluded that the second enzyme responsible for the degradation of 2-C-4-NA is a type of dioxygenase.

**Table 1:** Determination of aniline dioxygenase activity in strain MB-P1 measured by oxygen uptake by 2-C-4NA-grown versus 1/4-NB-grown cells^a^.

Substrates	O_2_ uptake (nmol O_2_/min/mg of protein) by cells grown in:	
	2-C-4-NA	1/4-NB
2-Chloro-4-nitroaniline	90.17±0.5	38.43±0.8
4-Amino-3-chlorophenol	59.70±1.5	0.15±0.2
4-Nitroaniline	83.13±0.2	42.41±1.0
4-Chloroaniline	69.10±0.8	23.35±0.1
Aniline	53.3±1.3	0.13±0.3

a The reaction was carried in 1.85 ml volume air-saturated phosphate buffer (20 mM, pH 7.2) containing substrates (40 µM), and cells (0.25 mg of protein). Data represents means of at least three separate experiments.

### Ring cleavage inhibition studies

The HPLC analysis of the samples collected from the ring cleavage inhibition studies by 2, 2-dipyridyl on 2-C-4-NA showed the accumulation of 6-CHQ at the R*t* value of 3. 28 minute with the liberation of only NO_2_^−^ ions and NH_3_ in the culture media (Figure 4A). The culture media became deep red in color, which also indicates accumulation of hydroxyquinol as reported previously [27], [35]. Noticeably, a slight accumulation of 6-CHQ in the control (without added 2, 2-dipyridyl) was observed which got disappeared within a short time of incubation with the liberation of NO_2_^−^, Cl^−^ ions, and NH_3_ (Figure 4B). The above results clearly suggested that 6-CHQ is the terminal intermediate for the degradation of 2-C-4-NA by strain MB-P1. It is well known that the reaction mechanism of 2, 2-dipyridyl used as an inhibitor for the ring cleavage require ferrous ions for their enzymatic activities [21]. The formation of hydroxyquinol as a terminal ring cleavage substrate has been exclusively reported in the degradation pathway of 4-nitrophenol by gram-positive bacteria [35]–[37]. Similarly, the formation of 6-chlorohydroxyquinol has also been reported as a ring cleavage substrate in the degradation pathway of 4-chlorophenol [21]. Based on the identified metabolite from the resting cell study, oxygen uptake, enzyme assays and ring cleavage inhibition study, the pathway for the degradation of 2-C-4-NA has been proposed as shown in Figure 5.

**Figure 4:** Ring cleavage inhibition studies using 2, 2-dipyridyl. (A) Treated with 2, 2-dipyridyl. (B) Untreated with 2, 2-dipyridyl. 2-C-4-NA (•); 4-A-3-CP (▴); and 6-CHQ (○).Values are presented as arithmetic means of data obtained from experiments carried out in triplicates; error bars represent standard deviation.

**Figure 5:** Proposed metabolic pathway for aerobic degradation of 2-C-4-NA by *Rhodococcus* sp. strain MB-P1. According to the results obtained presented here, 4-A-3-CP and 6-CHQ are identified as major intermediates during degradation of 2-C-4-NA.

## Discussion

Biodegradation has been recognized as an economical and environment friendly approach for decontamination of sites polluted with toxic anthropogenic chemicals, released into environment as a result of industrial, agricultural, military and household activities [38], [39]. Conversely, its application has remained elusive and inefficient in case of highly recalcitrant compounds including chloro and nitro containing anilines [14], [40], [41]. To overcome this limitation, it is essential to isolate and characterize microorganism(s) with potential to metabolize these compounds. To date no aerobic degradation and pathway characterization has been reported for the microbial degradation of 2-C-4-NA. However, based on the earlier reports on the degradation of structural analogues of 2-C-4-NA such as anilines substituted with chloro and nitro groups, it is presumed that the degradation of 2-C-4-NA could also be possible in aerobic condition. Although, the enrichment of cultures could be used as an efficient approach for isolating microorganism(s) with desired degradative capabilities; however, determining metabolic diversity of naturally occurring degradative isolates could also be another approach. Results presented in few recent studies indicate some degradative strains to be metabolically versatile that they can degrade compounds analogous to their original enrichment substrate. The genus of *Rhodococcus* constitutes a diverse group of bacteria which exhibit a metabolic versatile activity on chloro and nitro substituted aromatic compounds [42]. The catabolic versatility of *Rhodococcus* is due to the presence of large genome and plasmid which harbors large number of metabolic genes, resulting in expansion of the multiple metabolic pathways [43]. Ghosh and co-workers reported *Rhodococcus imtechiensis* strain RKJ300 with the ability to degrade 4-nitrophenol, 2, 4-dinitrophenol as well as their chloro substituted analogue 2-chloro-4-nitrophenol [42]. Based on the above rationale, the screening for the degradation of 2-C-4-NA was performed by using previous lab isolates known for the degradation of nitroaromatic compounds. The 2-C-4-NA degrading abilities were examined by analyzing the increase in growth and also by measuring the release of NO_2_^−^, Cl^−^, and NH_3_ in the medium. Results from primary screening, five strains belonging to the genus *Rhodococcus* showed the apparent increase of bacterial cell mass as well as the release of NO_2_^−^, Cl^−^ ions, and NH_3_. All these five isolates have been previously characterized for the degradation of chloro and nitro substituted aromatic compounds. Interestingly, the strain MB-P1 showed the faster degradation of 2-C-4-NA, hence it was selected for the detailed study. During the growth study, the rapid disappearance of 2-C-4-NA was accompanied by the release of NO_2_^−^ ions and NH_3_ followed by the release of Cl^−^ ions in the media. The amounts of chloride and nitrite ions accumulated in growth media were stoichiometric; however, very limited amounts of NH_3_ was released. There was no accumulation of intermediates of 2-C-4-NA degradation in the growth study. Based on the growth study it could be argued that 2-C-4-NA was completely mineralized and NH_3_ is the preferred nitrogen source for the growth of strain MB-P1. The above results are in close agreement with the results of 5-nitroanthranilic acid degradation by *Bradyrhizobium* sp. strain JS329 [44]. Although, the growth study did not show any accumulation of metabolites, however, the resting cell studies showed the formation of 4-A-3-CP as the first intermediate, which subsequently disappeared with the formation of 6-CHQ as a second metabolite. Results from elucidation of the catabolic pathway in 2-C-4-NA degradation by strain MB-P1 clearly demonstrated identification of 4-A-3-CP and 6-CHQ as major intermediates. There are two ways for the removal of nitro group from the chloronitrobenzenes or chloronitrophenols out of which one is oxidative and another one is reductive reaction mechanism. In the oxidative reaction the nitro group is removed in the form of NO_2_^−^ ions as a results of hydroxylation, while a partial reduction of nitro group into hydroxylamine or amino group takes place in reductive reaction [42], [45]–[49]. Results showing transformation of 2-C-4-NA to 4-A-3-CP for initiation of 2-C-4-NA degradation by strain MB-P1 suggest the involvement of oxygenation reaction by a putative monooxygenase. The monooxygenase enzyme assays from the crude cell extracts confirm the involvement of flavin-dependent monooxygenase. The flavin-dependent monooxygenase reaction is very common for aerobic microbial degradation of nitro or chloro containing aromatic compounds such as 2-chloro-4-nitrophenol, 4-nitrophenol, 2,4-dichlorophenol and 4-chlorophenol by aerobic microorganisms [42], [50]–[51]. In the proposed pathway, conversion of 4-A-3-CP into 6-CHQ is expected to be catalyzed by an enzyme capable of removing amino group via oxidative reaction. Mostly the removal of amino group from the benzene ring occurs by the action of catechol dioxygenase [44]. Such catalytic reaction mechanisms are widely distributed among the microorganisms capable of degrading anilines and chloroanilines [22], [33], [40], [52]–[55].

These microorganisms utilize aniline as the sole carbon, nitrogen, and energy source and degradation occurs via the formation of catechol metabolite with the action of catechol dioxygenase [22], [56]–[60]. Schukat et al. [61] reported the co-metabolic degradation of chloroanilines by *Rhodococcus* sp. An117 via the formation of catechol as terminal intermediate. Similarly, Zeyer et al. [62] reported utilization of chloroaniline by *Moraxella* sp. strain G occurs by *ortho-*pathway. Thus, the enzyme which is involved in the second step degradation of 2-C-4-NA i. e. conversion of 4-A-3-CP to 6-CHQ should be almost similar with those responsible for aniline and chloroaniline catabolism. The identified metabolite 6-CHQ from the resting cell study constitute the ring cleavage substrate during the 2-C-4-NA degradation by *Rhodococcus* sp. strain MB-P1 as supported by the accumulation of 6-CHQ during the ring cleavage inhibition study. The above result is in close agreement with results reported for 4-chlorophenol degradation by *Arthrobacter chlorophenolicus* A6 [27]. Based on such reports as well as the results obtained during the present study, we propose the possible involvement of a similar bacterial monooxygenase in the first step of 2-C-4-NA degradation followed by aniline dioxygenase mediated reaction as the second step of degradation. Subsequent degradation of terminal intermediate 6-CHQ presumably proceeds via conventional 2, 4, 6-trichlorophenol degradation pathway.

### Conclusion

In conclusion, we report metabolism of 2-C-4-NA by *Rhodococcus* sp. strain MB-P1 which was previously characterized for atrazine degradation. This is one of the first aerobic bacteria capable of degrading 2-C-4-NA as the sole carbon, nitrogen, and energy source. Strain MB-P1 degrades 2-C-4-NA via the formation of 4-A-3-CP and 6-CHQ as the novel intermediates. The first step of 2-C-4-NA degradation occurs by flavin-dependent monooxygenase mediated reaction with the formation of 4-A-3-CP which gets subsequently transformed to 6-CHQ via dioxygenation reaction. The lack of induction period and accumulation of 4-A-3-CP metabolite during the induction study of 2-C-4-NA degradation by strain MB-P1 confirmed the constitutive activity of first enzyme i. e. flavin-dependent monooxygenase. The above results were also supported by the results of oxygen uptake. However, the second enzyme responsible for the conversion of 4-A-3-CP to 6-CHQ is inducible in nature as confirmed from the oxygen uptake and induction studies. Strain MB-P1 could be used as a model system for studies focusing on this important transformation reaction for the degradation of chloro and nitro group containing anilines. Strain MB-P1 could also be used as an important model system for studies on biochemical and molecular evolution of microbial degradation of 2-C-4-NA. From application point of view, strain MB-P1 could be potentially used for bioremediation of ecological niches contaminated with 2-C-4-NA. The molecular components involved in the pathway of 2-C-4-NA degradation by strain MB-P1 are yet to be characterized.
